This article has been retracted.

# Post-operative blood pressure and 3-year major adverse cardiac events in Chinese patients undergoing PCI

**DOI:** 10.1186/s12872-021-02435-2

**Published:** 2021-12-30

**Authors:** Lijun Gan, Dandan Sun, Yuntao Cheng, Deyang Wang, Fen Wang, Lin Wang, Wei Li, Dandan Shen, Daotong Guo, Zonglei Zhang, Haiyan Wang, Jinli Li, Yong Yang, Tao Liang

**Affiliations:** 1 Department of Cardiology, Affiliated Hospital of Jining Medical University, Jining, Shandong China; 2 Cardiac Emergency Department, Affiliated Hospital of Jining Medical University, Jining, Shandong China; 3 Catheterization Room, Affiliated Hospital of Jining Medical University, Jining, Shandong China; 4 Department of Nursing, Affiliated Hospital of Jining Medical University, Jining, Shandong China; 5 School of Nursing, Peking Union Medical College, Beijing, China

## Abstract

**Background:**

There is no clear evidence for the target value of blood pressure control after Percutaneous coronary intervention (PCI). Therefore, our study was designed to explore the relationship between blood pressure after PCI and major adverse cardiac events (MACE) during 3-year follow-up.

**Methods:**

This study is a prospective study. We included the patients who were diagnosed with acute coronary syndrome and underwent PCI stent implantation operation. The study initially collected information of 552 patients. The start and end times of the study are from January 1, 2017 to December 31, 2020. The independent variables of this study are the average systolic blood pressure and the average diastolic blood pressure after PCI. The dependent variable is the occurrence of MACE events in patients within 3 years after PCI. MACE is defined as acute myocardial infarction, recurring chest pain, heart failure, stroke, revascularization and cardiac death.

**Results:**

A total of 514 subjects met the inclusion criteria. The average age of the study subjects is 61.92 ± 9.49 years old, of which 67.12% are male. 94 subjects had a MACE event within 3 years, and the occurrence rate was 18.29%. There is no significant non-linear or linear relationship between diastolic blood pressure and MACE events. There is a curvilinear relationship between the average systolic blood pressure of patients after PCI and MACE events within 3 years and the inflection point is 121. On the left side of the inflection point, the effect size and 95% CI are 1.09 and 1.01–1.18, respectively (*P* = 0.029). The impact size and 95% CI at the right inflection point were 1.00 and 0.98–1.02(*P* = 0.604), respectively.

**Conclusion:**

There is a curvilinear relationship between systolic blood pressure and prognosis of patients after PCI. Under the premise of ensuring the safety of patients, maintaining lower blood pressure after surgery is beneficial to improve the prognosis of patients.

## Introduction

Hypertension is one of the important risk factors of coronary atherosclerosis [1–3]. The guidelines recommend that the blood pressure of patients with hypertension should be strictly controlled [4, 5]. It has long been believed that higher blood pressure will lead to higher mortality [6, 7], stroke [8–10] incidence and other cardiovascular adverse events [11]. The J-curve or U-curve relationship between blood pressure and adverse events has been verified in patients with heart failure, stable angina and hypertension [12–15]. At the same time, the time of blood pressure measurement in previous studies was mostly on admission, pre-procedural or during follow-up [16–18]. Percutaneous coronary intervention (PCI) is an important treatment for patients with acute coronary syndrome [19, 20]. We believe that the control of blood pressure after PCI is of great significance to improve the clinical outcome of patients. However, there is no clear evidence for the target value of blood pressure control within short term after stent implantation. In addition, there are racial differences between the Asian population and the Western population [21]. There is currently no research evidence about the correlation between blood pressure and clinical prognosis in Chinese patients after PCI. Therefore, our study was designed to explore the relationship between blood pressure after PCI and major adverse cardiac events (MACE) during 3-year follow-up.

## Participants and methods

### Study design

This study is a prospective study. The purpose of this study is to explore the relationship between the systolic and diastolic blood pressure after surgery and the occurrence of MACE events within 3 years of patients undergoing PCI in China. The independent variables of this study are the average systolic blood pressure and the average diastolic blood pressure after PCI.

### Participants

The patients in this study were non-selectively and consecutively collected from patients who were diagnosed with acute coronary syndrome and underwent PCI stent implantation operation from January to December 2017 in the Affiliated Hospital of Jining Medical University, Jining City, Shandong province, China. The information obtained by the research does not contain the patients’ private data. All patients participating in the study signed the study informed consent form. This study was approved by the Medical Science Research Ethics Committee of the Affiliated Hospital of Jining Medical University (Ethics Number: 2021C030).

The study initially collected information of 552 patients. The start and end times of the study are from January 1, 2017 to December 31, 2020. The inclusion criteria were: (1) the patients who were diagnosed with acute coronary syndrome; (2) the patient underwent PCI stent implantation operation. The exclusion criteria were: (1) the patients who lost in follow-up due to change of mobile phone number, refused to answer the phone or other reasons; (2) death in the hospital; (3) the patient refused to answer questions during the follow-up process and withdrew from the study.

### Variables

We collected the blood pressure values of patients after PCI and recorded them as continuous variables. We recorded the patient's blood pressure 9 times, including immediately after surgery, 30 min after surgery, 1 h after surgery, 1.5 h after surgery, 2 h after surgery, 4 h after surgery, 6 h after surgery, 12 h after surgery, and 24 h after surgery. We calculate the average value of the patient's 9 systolic and diastolic blood pressures as the independent variable of this study. The blood pressure of the patients was measured with a Mindray ECG monitor. Before the measurement, keep the patient in a quiet state for 10–20 min, and prohibit smoking, tea and coffee. All of the patients wear the same uniform and measure the left upper extremity. During the measurement, the patient was placed in a supine position and align with the fourth intercostal space.

The dependent variable of this study is a binary variable. According to previous studies, we regard the occurrence of MACE within 3 years as the clinical outcome of the patient. The definition of MACE events in this study is as follows: follow-up by telephone and ask patients whether they have acute myocardial infarction, recurring chest pain, heart failure, stroke, revascularization, and cardiac death within 3 years after discharge. MACE events were first reported by the patients through telephone follow-up by the researchers. Then we identify the MACE event type through the medical system records. If any of the above outcomes occur, it is deemed that the patient has had a MACE event.

The variables included in this study include the following three aspects: (1) socio-demographic data of the subjects; (2) variables that may be related to MACE or blood pressure; and (3) other variables collected based on our clinical experience. Therefore, we used the following variables to construct a fully adjusted model: (1) the categorical variables included sex, smoking history, drinking history, education level, atrial fibrillation, diabetes, heart failure, myocardial infarction, myocardial bridge, cerebral infarction, number of stents implanted and medication after discharge; (2) continuous variable: body mass index (BMI), Cl^−^, Creatinine, Cysteine protease inhibitor C, free triiodothyronine (FT3), Free thyroxine (FT4), Thyroid Stimulating Hormone (TSH), high-density lipoprotein cholesterol (HDL-C), low-density lipoprotein cholesterol (LDL-C), Lipoprotein, K^+^, left ventricular ejection fraction (LVEF), Na^+^, total cholesterol (TC), triglyceride (TG), uric acid (UA)and urea.

### Follow-up procedure

The follow-up method in this study was telephone follow-up. The outcome of the MACE event was determined by the patients’ self-report. The follow-up was carried out by 5 members of the research group who had received standardized training. This study was followed up for 3 years. During the three-year period, follow-up visits were made every year.

### Statistical analysis

The continuous variables in accordance with the normal distribution are expressed by the mean ± standard deviation. The continuous variable of the skewness distribution is expressed by the median (minimum, maximum). Classification variables are expressed in frequency or percentage. We used χ^2^ (classified variable), one-way ANOVA test (normal distribution) or Kruskal-Whllis H test (skewness distribution) to test the differences of systolic blood pressure and diastolic blood pressure among three groups. The data analysis process of this study is based on three aspects: (1) the relationship between blood pressure and MACE events in patients after PCI (linear or nonlinear); (2) which factors interfere with the relationship between blood pressure and MACE events in patients after PCI; (3) what is the real relationship between blood pressure and MACE events in patients after PCI after stratified analysis. Therefore, the data analysis in this study is divided into two steps. Step 1: univariate and multivariate bivariate logistic regression were used. We build three models: model 1, a crude model with no covariates adjusted; model 2, adjusted social demographic data; and model 3, adjusted social demographic data and other covariables that may affect MACE events. Step 2: explain the nonlinear relationship between blood pressure and the occurrence of 3-year MACE events. Cox proportional hazard regression model using smooth curve fitting. If nonlinearity is detected, we first use a recursive algorithm to calculate the inflection point, and then construct a two-segment binary logic regression on both sides of the inflection point. Finally, the logarithmic likelihood ratio test is mainly used to determine which model is more suitable to fit the correlation between the target independent variable and the result variable. For continuous variables, we first convert them into classified variables according to tangent points. The likelihood ratio test was carried out after the effect adjustment test of the subgroup index. In order to ensure the robustness of data analysis, we carried out sensitivity analysis. We convert blood pressure into classification variables and calculate the *P* value of the trend. The aim is to verify the results of blood pressure as a continuous variable and to observe the possibility of nonlinearity. All the analyses were conducted using statistical software packages R (http://www.R-project.org, R Foundation) and EmpowerStats (http://www.empowerstats.com, X & Y Solutions, Inc, MA, USA). *P* values less than 0.05 (two-sided) were considered statistically significant.

## Results

### Baseline characteristics of selected participants

A total of 514 subjects met the inclusion criteria (see Fig. 1 for a flow chart). Table 1 is the baseline characters of the participants which is based on different groups of the systolic blood pressure and diastolic blood pressure. The average age of the study subjects is 61.92 ± 9.49 years old, of which 67.12% are male. 94 subjects had a MACE event within 3 years, and the occurrence rate was 18.29%. 3 cardiogenic death, 4 acute myocardial infarction, 15 revascularization, 5 stroke, 8 heart failure, and 90 recurrent chest pain. The incidence of MACE in the low, medium, and high systolic blood pressure groups were 15.79%, 19.88% and 19.19% respectively. The incidence of MACE in the low, medium, and high diastolic blood pressure groups were 16.96%, 17.06% and 20.81% respectively. No statistically significant differences were detected in Alcohol consumption, Smoke, AF, DM, heart failure history, Myocardial bridge, number of stents, Cl-, creatinine, FT3, FT4, HDL-C, LDL-C, Lipoprotein, K + , LVEF, TC, TG, UA, Urea, ACEI, Aspirin, Nitrates among different SBP groups (*P* > 0.05). The group with the highest systolic blood pressure had the oldest average age, the highest incidence of myocardial infarction, the highest BMI, Cysteine protease inhibitor C, TSH, and Na^+^ values, but the lowest incidence of cerebral infarction. No statistically significant differences were detected in Sex, Alcohol consumption, Smoke, Degree of education, AF, DM, heart failure history, Myocardial bridge, number of stents, Cl−, creatinine, Cysteine protease inhibitor C, FTH, HDL-C, LDL-C, Lipoprotein, K + , LVEF, Na + , TC, TG, Urea, ACEI, Aspirin, b-blocker, Clopidogrel, Nitrates, Ticagrelor among different DBP groups (*P* > 0.05). The group with the highest diastolic blood pressure had the lowest average age, the highest incidence of myocardial infarction, and the highest BMI, TSH, and UA values.

**Fig. 1:** Inclusion/exclusion criteria of the patients

**Table 1:** Baseline characteristics of participants

Blood pressure tertiles (mmHg)	SBP				DBP			
	Low 84–118	Middle 119–133	High 134–168	P value*	Low 53–70	Middle 71–79	High 80–105	P value*
*N*	171	171	172		171	170	173	
Age	61.82 ± 10.34	60.44 ± 9.66	63.50 ± 8.16	0.022	64.14 ± 10.05	61.26 ± 9.50	60.39 ± 8.52	< 0.001
*Sex*				0.002				0.852
Male	126 (73.68%)	121 (70.76%)	98 (56.98%)		112 (65.50%)	116 (68.24%)	117 (67.63%)	
Female	45 (26.32%)	50 (29.24%)	74 (43.02%)		59 (34.50%)	54 (31.76%)	56 (32.37%)	
*Alcohol consumption*				0.350				0.221
Nondrinker	105 (61.40%)	100 (58.48%)	113 (65.70%)		116 (67.84%)	104 (61.18%)	98 (56.65%)	
Current drinker	51 (29.82%)	62 (36.26%)	48 (27.91%)		45 (26.32%)	52 (30.59%)	64 (36.99%)	
Quit	15 (8.77%)	9 (5.26%)	11 (6.40%)		10 (5.85%)	14 (8.24%)	11 (6.36%)	
*Smoke or not*				0.288				0.718
Nonsmoker	82 (47.95%)	83 (48.54%)	97 (56.40%)		88 (51.46%)	83 (48.82%)	91 (52.60%)	
Current smoker	53 (30.99%)	61 (35.67%)	48 (27.91%)		53 (30.99%)	60 (35.29%)	49 (28.32%)	
Quit	36 (21.05%)	27 (15.79%)	27 (15.70%)		30 (17.54%)	27 (15.88%)	33 (19.08%)	
*Degree of education*				0.032				0.697
Illiterate	29 (16.96%)	38 (22.22%)	52 (30.23%)		43 (25.15%)	37 (21.76%)	39 (22.54%)	
Primary school	45 (26.32%)	34 (19.88%)	45 (26.16%)		46 (26.90%)	40 (23.53%)	38 (21.97%)	
Junior school	52 (30.41%)	56 (32.75%)	36 (20.93%)		48 (28.07%)	48 (28.24%)	48 (27.75%)	
High school and above	45 (26.32%)	43 (25.15%)	39 (22.67%)		34 (19.88%)	45 (26.47%)	48 (27.75%)	
*AF*				0.659				0.470
No	165 (96.49%)	167 (97.66%)	165 (95.93%)		167 (97.66%)	165 (97.06%)	165 (95.38%)	
Yes	6 (3.51%)	4 (2.34%)	7 (4.07%)		4 (2.34%)	5 (2.94%)	8 (4.62%)	
*DM*				0.876				0.766
No	125 (73.10%)	121 (70.76%)	125 (72.67%)		120 (70.18%)	125 (73.53%)	126 (72.83%)	
Yes	46 (26.90%)	50 (29.24%)	47 (27.33%)		51 (29.82%)	45 (26.47%)	47 (27.17%)	
*Heart failure history*				0.239				0.332
No	166 (97.08%)	170 (99.42%)	170 (98.84%)		168 (98.25%)	166 (97.65%)	172 (99.42%)	
Yes	5 (2.92%)	1 (0.58%)	2 (1.16%)		3 (1.75%)	4 (2.35%)	1 (0.58%)	
*Unstable angina*				< 0.001				< 0.001
No	108 (63.16%)	65 (38.01%)	35 (20.35%)		94 (54.97%)	60 (35.29%)	54 (31.21%)	
Yes	63 (36.84%)	106 (61.99%)	137 (79.65%)		77 (45.03%)	110 (64.71%)	119 (68.79%)	
*Myocardial infarction*				< 0.001				< 0.001
No	63 (36.84%)	106 (61.99%)	137 (79.65%)		77 (45.03%)	110 (64.71%)	119 (68.79%)	
Yes	108 (63.16%)	65 (38.01%)	35 (20.35%)		94 (54.97%)	60 (35.29%)	54 (31.21%)	
*Myocardial bridge*				0.398				0.124
No	161 (94.15%)	163 (95.32%)	157 (91.28%)		159 (92.98%)	155 (91.18%)	167 (96.53%)	
Yes	10 (5.85%)	8 (4.68%)	15 (8.72%)		12 (7.02%)	15 (8.82%)	6 (3.47%)	
*Cerebral infarction*				0.002				0.065
No	153 (89.47%)	149 (87.13%)	132 (76.74%)		152 (88.89%)	144 (84.71%)	138 (79.77%)	
Yes	18 (10.53%)	22 (12.87%)	40 (23.26%)		19 (11.11%)	26 (15.29%)	35 (20.23%)	
*Number of stent*				0.394				0.139
1	133 (77.77%)	123 (71.93%)	113 (65.69%)		136 (79.53%)	115 (67.65%)	118 (68.21%)	
2	26 (15.20%)	36 (21.05%)	45 (26.16%)		26 (15.20%)	44 (25.88%)	37 (21.39%)	
3	11 (6.43%)	10 (5.85%)	11 (6.40%)		8 (4.68%)	9 (5.29%)	15 (8.67%)	
4	1 (0.58%)	2 (1.17%)	3 (1.74%)		1 (0.58%)	2 (1.17%)	3 (1.73%)	
BMI	24.76 ± 3.53	25.83 ± 3.62	26.40 ± 3.68	< 0.001	24.72 ± 3.64	25.85 ± 3.31	26.41 ± 3.84	< 0.001
Cl^−^	102.33 ± 3.08	102.07 ± 3.17	102.72 ± 2.89	0.253	102.18 ± 3.08	102.42 ± 2.35	102.51 ± 3.58	0.496
Creatinine	67.42 ± 16.23	68.68 ± 24.28	69.93 ± 38.07	0.878	67.75 ± 17.27	68.50 ± 34.55	69.90 ± 29.47	0.788
Cysteine protease inhibitor C	1.05 ± 0.27	1.06 ± 0.30	1.15 ± 0.40	0.012	1.09 ± 0.27	1.09 ± 0.36	1.08 ± 0.37	0.563
FT3 Free triiodothyrotropin	4.61 ± 1.68	4.58 ± 0.78	4.93 ± 3.73	0.391	4.40 ± 0.96	5.05 ± 3.89	4.67 ± 1.27	0.039
FT4	16.50 ± 4.44	15.88 ± 2.17	16.46 ± 4.80	0.710	15.87 ± 2.62	16.56 ± 4.77	16.31 ± 3.97	0.940
TSH	2.11 ± 1.73	2.64 ± 1.82	3.71 ± 8.84	0.003	2.35 ± 2.02	2.34 ± 1.49	3.80 ± 8.74	0.016
HDL-C	1.08 ± 0.30	1.09 ± 0.27	1.07 ± 0.25	0.561	1.10 ± 0.30	1.07 ± 0.27	1.08 ± 0.24	0.925
LDL-C	2.42 ± 0.77	2.52 ± 0.85	2.53 ± 0.86	0.538	2.57 ± 0.92	2.48 ± 0.77	2.42 ± 0.80	0.612
Lipoprotein	182.00 (92.00–325.00)	169.50 (95.00–349.50)	190.50 (96.50–344.25)	0.848	218.00 (98.50–412.50)	157.00 (91.75–320.00)	165.00 (94.00–308.25)	0.120
K^+^	4.15 ± 0.42	4.22 ± 0.38	4.15 ± 0.44	0.226	4.18 ± 0.43	4.19 ± 0.43	4.16 ± 0.39	0.801
LVEF	55.66 ± 7.44	57.54 ± 5.35	57.90 ± 4.17	0.165	56.55 ± 6.56	57.24 ± 5.72	57.56 ± 4.91	0.632
Na^+^	140.83 ± 2.84	141.23 ± 2.84	141.81 ± 2.39	0.017	140.98 ± 2.84	141.49 ± 2.55	141.44 ± 2.74	0.143
TC	4.12 ± 1.08	4.29 ± 1.10	4.40 ± 1.14	0.091	4.34 ± 1.25	4.27 ± 1.03	4.21 ± 1.05	0.942
TG	1.50 ± 0.91	1.53 ± 1.00	1.72 ± 1.12	0.141	1.52 ± 1.05	1.60 ± 1.04	1.63 ± 0.96	0.350
UA	288.93 ± 90.22	308.09 ± 71.10	298.71 ± 78.67	0.112	294.57 ± 90.00	291.34 ± 74.43	310.63 ± 74.28	0.036
Urea	5.28 ± 1.78	5.40 ± 1.64	5.55 ± 2.03	0.317	5.48 ± 1.80	5.42 ± 2.05	5.34 ± 1.60	0.814
*ACEI*				0.178				0.584
No	109 (63.74%)	110 (64.33%)	124 (72.09%)		110 (64.33%)	118 (69.41%)	115 (66.47%)	
Yes	62 (36.26%)	61 (35.67%)	48 (27.91%)		61 (35.67%)	52 (30.59%)	58 (33.53%)	
*ARB*				< 0.001				< 0.001
No	159 (92.98%)	143(83.63%)	120 (69.77%)		159 (92.98%)	135 (79.41%)	128 (73.99%)	
Yes	12 (7.02%)	28 (16.37%)	52 (30.23%)		12 (7.02%)	35 (20.59%)	45 (26.01%)	
*Aspirin*				0.643				0.549
No	4(2.34%)	1 (0.58%)	3 (1.74%)		4 (2.34%)	3 (1.76%)	1 (0.58%)	
Yes	167 (97.66%)	170 (99.42%)	169 (98.26%)		167 (97.66%)	167 (98.24%)	172 (99.42%)	
*b-blocker*				0.019				0.921
No	24 (14.04%)	37 (21.64%)	44 (25.58%)		37 (21.64%)	33 (19.41%)	35 (20.23%)	
Yes	147 (85.96%)	134 (78.36%)	128 (74.42%)		134 (78.36%)	137 (80.59%)	138 (79.77%)	
*Clopidogrel*				0.043				0.321
No	83 (48.54%)	70 (40.94%)	60 (34.88%)		79 (46.20%)	65 (38.24%)	69 (39.88%)	
Yes	88 (51.46%)	101 (59.06%)	112 (65.12%)		92 (53.80%)	105 (61.76%)	104 (60.12%)	
*Nitrates*				0.587				0.265
No	71 (41.52%)	75 (43.86%)	66 (38.37%)		70 (40.94%)	63 (37.06%)	79 (45.66%)	
Yes	100 (58.48%)	96 (56.14%)	106 (61.63%)		101 (59.06%)	107 (62.94%)	94 (54.34%)	
*Stain*				0.007				0.035
No	10 (5.85%)	2 (1.17%)	1 (0.58%)		9 (5.26%)	1 (0.59%)	3 (1.73%)	
Yes	161 (94.15%)	169 (98.83%)	171 (99.42%)		162 (94.74%)	169 (99.41%)	170 (98.27%)	
*Ticagrelor*				0.029				0.363
No	95 (55.56%)	107 (62.57%)	119 (69.19%)		100 (58.48%)	109 (64.12%)	112 (64.74%)	
Yes	76 (44.44%)	64 (37.43%)	53 (30.81%)		71 (41.52%)	61 (35.88%)	61 (35.26%)	
*MACE*				0.577				0.574
No	144 (84.21%)	137 (80.12%)	139 (80.81%)		142 (83.04%)	141 (82.94%)	137 (79.19%)	
Yes	27 (15.79%)	34 (19.88%)	33 (19.19%)		29 (16.96%)	29 (17.06%)	36 (20.81%)	

### Result of univariate analysis

We listed the results of univariate analyses in Table 2. By univariate binary logistic regression, we found that age (1.03, 1.01–1.05), DM (2.01, 1.82–2.20), Cerebral infarction (1.85, 1.62–2.08) were positively correlated with the occurrence of MACE. LVEF (0.97, 0.95–0.99) was negatively associated with the occurrence of MACE.

**Table 2:** Univariate analysis for MACE of PCI patients

Covariate	Statistics	β (95%CI)	*P* value
Age	61.92 ± 9.49	1.03 (1.01, 1.05)	0.045
*Sex*			
Male	345 (67.12%)	Reference	
Female	169 (32.88%)	0.88 (0.54, 1.45)	0.625
*Alcohol consumption*			
Nondrinker	318 (61.87%)	Reference	
Current drinker	161 (31.32%)	0.94 (0.53, 1.66)	0.832
Quit	35 (6.81%)	0.54 (0.17, 1.66)	0.281
*Smoke or not*			
Nonsmoker	262 (50.97%)	Reference	
Current smoker	162 (31.52%)	1.08 (0.58, 2.02)	0.801
Quit	90 (17.51%)	1.00 (0.48, 2.06)	0.996
*Degree of education*			
Illiterate	119 (23.15%)	Reference	
Primary school	124 (24.12%)	1.69 (0.85, 3.35)	0.136
Junior school	144 (28.02%)	1.07 (0.50, 2.29)	0.868
High school and above	127 (24.71%)	1.54 (0.72, 3.27)	0.262
*AF*			
No	497 (96.69%)	Reference	
Yes	17 (3.31%)	0.48 (0.10, 2.21)	0.346
*DM*			
No	371 (72.18%)	Reference	
Yes	143 (27.82%)	2.01 (1.82, 2.20)	0.024
*Heart failure history*			
No	506 (98.44%)	Reference	
Yes	8 (1.56%)	0.64 (0.08, 5.32)	0.675
*Unstable angina*			
No	208 (40.47%)	Reference	
Yes	306 (59.53%)	1.24(0.78,1.98)	0.359
*Myocardial infarction*			
No	306 (59.53%)	Reference	
Yes	208 (40.47%)	0.90 (0.56, 1.46)	0.677
*Myocardial bridge*			
No	481 (93.58%)	Reference	
Yes	33 (6.42%)	0.84 (0.31, 2.25)	0.722
*Cerebral infarction*			
No	434 (84.44%)	Reference	
Yes	80 (15.56%)	1.85 (1.62, 2.08)	0.038
*Number of stent*			
1	369 (71.90%)	Reference	
2	107 (20.82%)	0.82 (0.46, 1.46)	0.499
3	32 (6.23%)	1.44 (0.62, 3.34)	0.401
4	6 (1.17%)	0.78 (0.09, 6.79)	0.819
BMI	25.67 ± 3.66	1.03 (0.97, 1.10)	0.384
Cl^−^	102.38 ± 3.05	1.00 (0.92, 1.08)	0.957
Creatinine	68.73 ± 28.04	1.00 (0.99, 1.01)	0.528
Cysteine protease inhibitor C	1.09 ± 0.34	1.19 (0.59, 2.39)	0.632
FT3 Free triiodothyrotropin	4.71 ± 2.43	0.92 (0.71, 1.18)	0.503
FTH Free thyroxine	16.25 ± 3.91	1.02 (0.95, 1.08)	0.605
TSH	2.87 ± 5.46	0.99 (0.93, 1.06)	0.756
HDL-C	1.08 ± 0.27	1.11 (0.43, 2.90)	0.827
LDL-C	2.49 ± 0.83	0.80 (0.59, 1.10)	0.178
Lipoprotein	179.00 (93.00–342.00)	1.00 (1.00, 1.00)	0.206
K^+^	4.17 ± 0.41	0.77 (0.42, 1.41)	0.396
LVEF	57.16 ± 5.70	0.97 (0.95, 0.99)	0.036
Na^+^	141.31 ± 2.71	0.97 (0.88, 1.06)	0.466
TC	4.27 ± 1.11	0.92 (0.72, 1.17)	0.495
TG	1.58 ± 1.02	1.08 (0.85, 1.37)	0.513
UA	298.99 ± 80.09	1.00 (1.00, 1.00)	0.294
Urea	5.41 ± 1.82	1.09 (0.96, 1.24)	0.194
*ACEI*			
No	343 (66.73%)	Reference	
Yes	171 (33.27%)	0.95 (0.58, 1.55)	0.834
*ARB*			
No	422 (82.10%)	Reference	
Yes	92 (17.90%)	1.44 (0.84, 2.48)	0.190
*Aspirin*			
No	8 (1.56%)	Reference	
Yes	506 (98.44%)	1.10 (0.13, 9.39)	0.934
*b-blocker*			
No	105(20.43%)	Reference	
Yes	409 (79.57%)	1.45 (0.79, 2.68)	0.232
*Clopidogrel*			
No	213 (41.44%)	Reference	
Yes	301 (58.56%)	0.67 (0.42, 1.06)	0.087
*Nitrates*			
No	212 (41.25%)	Reference	
Yes	302 (58.75%)	1.08 (0.66, 1.75)	0.756
*Stain*			
No	13 (2.53%)	Reference	
Yes	501 (97.47%)	0.95 (0.20, 4.47)	0.945
*Ticagrelor*			
No	321 (62.45%)	Reference	
Yes	193 (37.55%)	1.41 (0.88, 2.25)	0.155

### Results of unadjusted and adjusted binary logistic regression

In this study, we constructed three models to verify the relationship between systolic or diastolic blood pressure and the occurrence of MACE events respectively. The specific values of the effect size and 95% confidence interval are shown in Tables 3 and 4. In the crude model, the model-based effect size can be interpreted as a change in the risk of a MACE event for every unit change in blood pressure. For systolic blood pressure, in the crude model and model 2, for 1 mmHg increase in systolic blood pressure, the risk of MACE events increases by 1% (1.01, 95% CI 1.00–1.03). In model 3, for 1 mmHg increase in systolic blood pressure, the risk of MACE events increases by 1% (1.01, 95% CI 0.99–1.03). For diastolic blood pressure, in the crude model, the occurrence of MACE events does not change with changes in diastolic blood pressure (1.00, 95% CI 0.98–1.03). In model 2, for 1 mmHg increase in diastolic blood pressure, the risk of MACE events increases by 1% (1.01, 95% CI 0.98–1.03). In Model 3, the occurrence of MACE events has no correlation with changes of DBP. We converted the blood pressure value into a categorical variable (Tertile of SBP and DBP) for the purpose of sensitivity analysis. We performed a trend test on the *P* value, and the results were consistent with the result when blood pressure as a continuous variable.

**Table 3:** Relationship between SBP and MACE in different models

Variable	Crude model (model 1)	Adjust I (model 2)	Adjust II (model 3)
SBP (mmHg)	1.01 (1.00, 1.03) 0.107	1.01 (1.00, 1.03) 0.125	1.01 (0.99, 1.03) 0.202
*SBP (mmHg) Tertile*			
84–118	Reference	Reference	Reference
119–133	1.32 (0.76, 2.31) 0.324	1.37 (0.78, 2.40) 0.271	1.27 (0.65, 2.48) 0.481
134–168	1.36 (0.78, 2.37) 0.274	1.33 (0.76, 2.33) 0.314	1.37 (0.70, 2.68) 0.362
*P* for trend	1.16 (0.88, 1.53) 0.279	1.15 (0.87, 1.51) 0.319	1.16 (0.83, 1.62) 0.374

All adjusted for age, sex, diabetes, cerebral infarction and LVEF

**Table 4:** Relationship between DBP and MACE in different models

Variable	Crude model (model 1)	Adjust I (model 2)	Adjust II (model 3)
DBP (mmHg)	1.00 (0.98, 1.03) 0.867	1.01 (0.98, 1.03) 0.601	1.00 (0.97, 1.03) 0.977
*DBP (mmHg) Tertile*			
53–70	Reference	Reference	Reference
71–79	1.01 (0.58, 1.76) 0.980	1.08 (0.61, 1.89) 0.800	0.83 (0.43, 1.61) 0.015
80–105	1.23 (0.72, 2.12) 0.442	1.35 (0.78, 2.34) 0.286	1.13 (0.60, 2.11) 0.713
*P* for trend	1.11 (0.85, 1.46) 0.436	1.16 (0.88, 1.53) 0.282	1.08 (0.78, 1.48) 0

All adjusted for age, sex, diabetes, cerebral infarction and LVEF

### Results of nonlinearity of blood pressure and MACE

In this study, we analyzed the non-linear relationship between the blood pressures of patients after PCI and the occurrence of MACE events within 3 years (Fig. 2 is systolic blood pressure, Fig. 3 is diastolic blood pressure). Smooth curve and the result of the Cox proportional hazards regression model with cubic spline functions showed that the relationship between systolic blood pressure and MACE was nonlinear after adjusting for age, sex, diabetes, cerebral infarction and LVEF.. We used both binary logistic regression and two-piecewise binary logistic regression to fit the association and select the best fit model based on *P* for the log likelihood ratio test.

**Fig. 2:** Association between systolic blood pressure and the occurrence of MACE

**Fig. 3:** Association between diastolic blood pressure and the occurrence of MACE

When we analyzed the relationship between diastole and MACE events, the log-likelihood ratio test *P* was greater than 0.05. This shows that there is no significant non-linear or linear relationship between diastolic blood pressure and MACE events. When analyzing the relationship between systolic blood pressure and MACE events, because the* P* of the log-likelihood ratio test is less than 0.05, we chose a two-part binary logistic regression to fit the relationship between systolic blood pressure and the occurrence of MACE events in 3 years. Through the two-part binary logistic regression and recursive algorithm, we calculated the inflection point was 121. On the left side of the inflection point, the effect size and 95% CI are 1.09 and 1.01–1.18, respectively (*P* = 0.029). The impact size and 95% CI at the right inflection point were 1.00 and 0.98–1.02 (*P* = 0.820), respectively (Table 5).

**Table 5:** Results of SBP and MACE using two piecewise linear regression

Inflection point of platelets	Effect size	95% CI	*P* value
< 121	1.09	1.01–1.18	0.029
≥ 121	1.00	0.98–1.02	0.820

## Discussion

Our study found that there is a curvilinear relationship between the average systolic blood pressure of patients after PCI and MACE events within 3 years. At the same time, we found the inflection point of systolic blood pressure at 121. On the left side of the inflection point, the effect size and 95% CI are 1.09 and 1.01–1.18, respectively (*P* = 0.029). The impact size and 95% CI at the right inflection point were 1.00 and 0.98–1.02, respectively (P = 0.820). Only to the left of the inflection point, there is a statistical correlation between systolic blood pressure and the occurrence of MACE events. In addition, we did not find a clear statistical correlation between the diastolic blood pressure and the occurrence of MACE events.

Josephine et al. [16] measured blood pressure before PCI and analyzed its influence on long-term prognosis. Their results showed that patients with higher pulse pressure had a worse prognosis, while patients with higher pulse pressure had higher systolic blood pressure. Josephine et al. believed that high systolic blood pressure leads to left ventricular hypertrophy, increased cardiac afterload, increased wall stress and myocardial oxygen consumption. Therefore, the prognosis of the patients with higher SBP is poor. This is consistent with our research results. Besides, Han Pan et al. [22] conducted a meta-analysis on blood pressure and sudden cardiac death in patients. The results of the study showed that there is a curvilinear relationship between SBP and sudden cardiac death. For per 20 mmHg increase in systolic blood pressure, the risk of sudden death in patients increased by 9%. This is consistent with the results of this study, that is, within a certain range, as the systolic blood pressure increases, the patient's prognosis is poor. Analyzing the reasons, this may be related to the following factors: (1) Increased systolic blood pressure leads to increased cardiac afterload, and myocardial oxygen consumption increases after PCI. The probability of recurrence of angina pectoris increases. (2) Patients with higher systolic blood pressure after PCI tend to have higher basal blood pressure, the patients tend to with chronic left ventricular hypertrophy. The left ventricular hypertrophy is one of the risk factors for ventricular arrhythmia [23, 24]. (3) Hypertension after PCI may lead to abnormal cardiac electrophysiology and changes in left atrial structure and function, which may lead to atrial fibrillation [25], which is closely related to the occurrence of heart failure and stroke.

Previous studies have not conducted relevant studies on blood pressure control in the short-term after PCI. However, previous studies have explored the relationship between the admission blood pressure of patients with myocardial infarction and the prognosis in the hospital. But there are some studies inconsistent with the results of our study. For example, Shiraish et al. [26] conducted a study on patients undergoing PCI with acute myocardial infarction in Japan and showed that admission of SBP 141–158 mmHg may be associated with better in-hospital prognosis. The admission SBP < 105 mmHg is associated with the death of PCI patients in the hospital. Hyukjin et al. [18] conducted a study on Korean patients with acute myocardial infarction and showed that there is a U-shaped curve between SBP and DBP and MACE events, with an average SBP of 112.2 mmHg, and the lowest incidence of MACE events during DBP. It is 73.3 mmHg. An analysis of the International Verapamil SRTrandolapril Study (INVEST) [27] suggested that the relation between MACE rate and SBP was J-shaped. Analysis of the reasons for the inconsistency between the above research and our research results may be as follows: (1) The blood pressure data collected in this study comes from the average value after PCI, not the blood pressure at admission. The results of this study prove that if the systolic blood pressure is too high after revascularization, it will lead to an increase in cardiac afterload. (2) Previous studies grouped blood pressure values into groups and analyzed them as categorical variables. Our research treats blood pressure as a continuous variable, which can more accurately explore the relationship between blood pressure and the occurrence of MACE events. (3) In previous studies, MACE events were measured in hospital or short-term follow-up, while our study was followed up for 3 years.

Our research has the following three advantages. First of all, our study provides the target direction for blood pressure control after PCI for the first time. Early postoperative blood pressure control is a key clinical concern for doctors and nurses. This is not explored in previous studies. Secondly, our research separately explored the curve relationship between systolic and diastolic blood pressure and long-term prognosis, and found the inflection point of systolic blood pressure. This has important guiding significance for clinical practice. Third, this observational study adjusted multiple confounding variables to more clearly describe the relationship between blood pressure and the long-term prognosis of patients after PCI.

However, our study also has some limitations. First of all, our research is only a single-center study, and the subjects are all from the same hospital in Shandong Province, China. Second, our study only explored the impact of blood pressure on the prognosis of patients after PCI. In the future, the blood pressure of patients after discharge can be monitored and observed to find the long-term blood pressure target value of patients after discharge, so that the patients can get the maximum benefit. At last, MACE events were first reported by the patients through telephone follow-up by the researchers. Then we identify the MACE event type through the medical system records. However, the possibility that the patient may seek treatment in other medical institutions cannot be ruled out. If the patient’s medical treatment information cannot be retrieved, the patient’s self-reported outcome shall prevail. This is also one of the limitations of this study.

## Conclusions

There is a curvilinear relationship between systolic blood pressure and prognosis of patients after PCI. Under the premise of ensuring the safety of patients, maintaining lower blood pressure after surgery is beneficial to improve the prognosis of patients. In the future, the blood pressure of patients after discharge can be monitored and observed to find the long-term blood pressure target value of patients after discharge, so that the patients can get the maximum benefit.

## Data Availability

For data sharing, please contact the corresponding author of this article.

## Abbreviations

PCI: Percutaneous coronary intervention
MACE: Major adverse cardiac events
BMI: Body mass index
FT3: Free triiodothyronine
FT4: Free thyroxine
TSH: Thyroid stimulating hormone
HDL-C: High-density lipoprotein cholesterol
LDL-C: Low-density lipoprotein cholesterol
LVEF: Left ventricular ejection fraction
TC: Total cholesterol
TG: Triglyceride
UA: Uric acid
